# Gene Expression Profiling of Type 2 Diabetes Mellitus by Bioinformatics Analysis

**DOI:** 10.1155/2020/9602016

**Published:** 2020-10-21

**Authors:** Huijing Zhu, Xin Zhu, Yuhong Liu, Fusong Jiang, Miao Chen, Lin Cheng, Xingbo Cheng

**Affiliations:** ^1^Department of Endocrinology and Metabolism, The First Affiliated Hospital of Soochow University, Suzhou, Jiangsu, China; ^2^Department of Endocrinology and Metabolism, Heze Municipal Hospital, Heze, Shandong, China; ^3^Department of Endocrinology and Metabolism, The Affiliated Sixth People's Hospital of Shanghai Jiao Tong University, Shanghai, China; ^4^Department of ICU, Heze Municipal Hospital, Heze, Shandong, China

## Abstract

**Objective:**

The aim of this study was to identify the candidate genes in type 2 diabetes mellitus (T2DM) and explore their potential mechanisms.

**Methods:**

The gene expression profile GSE26168 was downloaded from the Gene Expression Omnibus (GEO) database. The online tool GEO2R was used to obtain differentially expressed genes (DEGs). Gene Ontology (GO) term enrichment analysis and Kyoto Encyclopedia of Genes and Genomes (KEGG) pathway analysis were performed by using Metascape for annotation, visualization, and comprehensive discovery. The protein-protein interaction (PPI) network of DEGs was constructed by using Cytoscape software to find the candidate genes and key pathways.

**Results:**

A total of 981 DEGs were found in T2DM, including 301 upregulated genes and 680 downregulated genes. GO analyses from Metascape revealed that DEGs were significantly enriched in cell differentiation, cell adhesion, intracellular signal transduction, and regulation of protein kinase activity. KEGG pathway analysis revealed that DEGs were mainly enriched in the cAMP signaling pathway, Rap1 signaling pathway, regulation of lipolysis in adipocytes, PI3K-Akt signaling pathway, MAPK signaling pathway, and so on. On the basis of the PPI network of the DEGs, the following 6 candidate genes were identified: PIK3R1, RAC1, GNG3, GNAI1, CDC42, and ITGB1.

**Conclusion:**

Our data provide a comprehensive bioinformatics analysis of genes, functions, and pathways, which may be related to the pathogenesis of T2DM.

## 1. Introduction

Type 2 diabetes mellitus (T2DM), a disease with significant morbidity, disability, and mortality, has affected increasing numbers of people worldwide. The World Health Organization (WHO) projected that diabetes would be the 7th leading cause of death in 2030. In addition, it has been predicted that by 2030, developing countries would account for 77.6% of all diabetic patients [1]. Although diabetes is a chronic disease that often causes various complications, in terms of financial burden, the cost of diabetes is 2-4 times more than that of the average patient in all medical systems [2]. Early detection and diagnosis of diabetes to prevent diabetes-associated complications and to reduce the economic costs on medical care are therefore of significant importance.

T2DM, which is characterized by hyperglycemia in the case of insulin resistance and impaired insulin secretion, is also a multigene heterogeneous disease that is the result of the interaction of genetic and environmental factors [3]. Although genetic factors play an important role in the occurrence and development of T2DM, the elaboration of its exact mechanism depends on the identification of susceptibility genes for T2DM.

At present, most of the gene research on T2DM mainly uses gene chip technology to detect and analyze model animals or clinical patient samples alone. Through this single analysis method, some valuable genes can be screened out for research and analysis. Gene expression analysis based on microarray technology is a powerful and high-throughput research method. Through gene expression profiling, some studies have found that hundreds of differentially expressed genes (DEGs) are involved in multiple molecular functions, biological processes, and signaling pathways [4], which played an important role in the occurrence and development of diseases and could be used as a potential molecular target and diagnostic marker. In the current study, the GSE26168 dataset [5] was downloaded from the Gene Expression Omnibus (GEO) database to identify T2DM-associated DEGs between T2DM and normal samples. Subsequently, GO term enrichment analysis, Kyoto Encyclopedia of Genes and Genomes (KEGG) pathway analysis, and PPI network analysis were performed to discover candidate genes as T2DM biomarkers and therapeutic targets worthy of further progress.

## 2. Methods

### 2.1. Microarray Data

The dataset GSE26168 based on the GPL6883 platform (Illumina HumanRef-8 v3.0 expression bead chip) was downloaded from GEO. A total of 9 T2DM samples and 8 normal samples were analyzed.

### 2.2. Identification of DEGs

GEO2R (http://www.ncbi.nlm.nih.gov/geo/geo2r/) is an interactive web tool for comparing two sets of data under the same experimental conditions and can analyze any geo series [6]. GEO2R was applied to explore DEGs between T2DM and normal blood samples. Statistically significant DEGs were defined with ∣logFC | ≥2, and the *P* value < 0.05 was the cut-off criterion.

### 2.3. Functional and Pathway Enrichment Analysis of DEGs

GO is a common way to annotate genes, gene products, and sequences as potential biological phenomena, mainly including biological process (BP), cellular component (CC), and molecular function (MF); the Kyoto Encyclopedia of Genes and Genomes (KEGG) is a comprehensive database resource for the biological interpretation of genomic sequences and other high-throughput data. GO and KEGG analyses were performed using the Metascape database to analyze the DEGs at the functional level. A *P* value < 0.01 and min overlap > 3 were set as the cut-off criterion.

### 2.4. Integration of the Protein-Protein Interaction (PPI) Network

The PPI network of DEGs was constructed by STRING. A confidence score ≥ 0.9 was set as significant. Subsequently, the PPI networks were visualized using Cytoscape software (3.7.1). MCODE was used to screen out the core genes that constitute the stable structure of the PPI network with degree cut‐off = 3, haircut on, node score cut‐off = 0.2, *k*‐core = 4, and maximum depth = 100. Moreover, the CentiScape plug-in was used to calculate the centrality index and topological properties for the identification of the most important nodes of a network, including undirected, directed, and weighted networks. The key (hub) genes were defined with degree value ≥ mean + 2SD, while the bottleneck genes were defined with betweenness value ≥ mean + 2SD. Then, using Venn diagram analysis, the genes in the intersection of the above three datasets were selected as candidate genes for the diagnosis of T2DM.

## 3. Results

### 3.1. Identification of DEGs

Based on the aforementioned threshold (∣logFC | ≥2 and *P* < 0.05), a total of 981 DEGs including 301 upregulated DEGs and 680 downregulated DEGs were filtered with GEO2R (Figure 1).

### 3.2. Functional and Pathway Enrichment Analysis

Three GO category results are presented in Figures 2(a)–2(c). As to the biological process (BP), DEGs were significantly enriched in cell morphogenesis involved in differentiation, chemotaxis, and regulation of cell adhesion (Figure 2(a)). For the cell component (CC), DEGs were enriched in the microtubule organizing center, dendrite, and anchored component of the membrane (Figure 2(b)). In terms of the molecular function (MF), DEGs were enriched in protein domain-specific binding, ubiquitin protein ligase binding, and anion transmembrane transporter activity (Figure 2(c)). The KEGG pathway analysis revealed that DEGs were highly associated with the cAMP signaling pathway, Rap1 signaling pathway, and bacterial invasion of epithelial cells (Figure 3).

### 3.3. PPI Network Construction and Analysis of Modules

The PPI network consisted of 945 nodes and 835 edges after hiding nodes which could not interact with other nodes (Figure 4(a)). Then, we used MCODE to perform *K* kernel analysis of the string network, a total of 9 clusters were generated, and 90 core genes were screened out (Table 1, Figures 4(b)–4(j)). Besides, the topology characteristics of the string network and each node were computed with CentiScape. 12 hub genes and 14 bottleneck genes were obtained (Table 1). Moreover, using Venn diagram analysis, 6 candidate genes in the intersection of the above three datasets were selected for further analysis, including phosphoinositide-3-kinase regulatory subunit 1 (PIK3R1), ras-related C3 botulinum toxin substrate 1 (rho family, small GTP-binding protein Rac1) (RAC1), G protein subunit gamma 3 (GNG3), G protein subunit alpha i1 (GNAI1), cell division cycle 42 (CDC42), and integrin subunit beta 1 (ITGB1) (Figure 5).

## 4. Discussion

In this study, we identified a total of 981 significant DEGs between T2DM and normal samples, including 301 upregulated genes and 680 downregulated genes, and conducted a series of bioinformatics analysis to screen candidate genes and pathways related to T2DM. DEGs were investigated in both GO term enrichment analysis and KEGG pathway analysis for functional annotation. As the outcomes of GO term enrichment analysis, DEGs might play critical roles in T2DM through cell differentiation, cell adhesion, intracellular signal transduction, and regulation of protein kinase activity. Meanwhile, KEGG pathway analysis revealed that DEGs were mainly enriched in the cAMP signaling pathway, Rap1 signaling pathway, regulation of lipolysis in adipocytes, PI3K-Akt signaling pathway, and MAPK signaling pathway. Moreover, by constructing the PPI, 6 candidate genes were identified, which exerted a momentous effect on the T2DM initiation, progression, and intervention strategy from different sides, including PIK3R1, RAC1, GNG3, GNAI1, CDC42, and ITGB1. The regulatory network consisting of microRNAs (miRNAs), long noncoding RNA (lncRNA), and mRNAs has attracted increasing attention to elucidate the mechanism of action in various diseases. In this study, mirDIP and starBase were used to analyze and predict the upstream miRNA interacting with candidate genes and the upstream lncRNA interacting with miRNA. A total of 22 miRNAs and 5 lncRNA were screened, which may play crucial parts in the development of T2DM.

PIK3R1 encodes the p85*α* regulatory subunit of the phosphatidylinositol-3-kinase (PI3K), which connects firmly with the p110 catalytic subunit, and together, they form the PI3K protein. PI3K plays a key role in insulin signaling by binding to phosphorylated insulin receptor substrates (IRS), producing phosphatidylinositol-4,5-trisphosphate (PIP3), which then activates several downstream targets such as AKT serine-threonine kinase [7]. AKT regulates cell survival, growth, differentiation, glucose transporter type 4 (GLUT-4) trafficking, and glucose utilization [8]. Mouse studies have shown that mice lacking PIK3R1 display enhanced insulin sensitivity and glucose tolerance, due to an improved stoichiometry of the p85*α*/p110 complex for binding to IRS and enhanced insulin-stimulated Akt activity [9, 10]. The overexpression of p85*α* weakens signal transmission and causes insulin resistance by disrupting the activity of the p85*α*/p110 complex and the connection between PI3K and IRS [11, 12], which indicates that p85*α* subunits play a negative role in PI3K signaling downstream of the insulin receptor. Thus, PIK3R1 is a logical candidate gene involved in the development of T2DM. Regulation of p85*α* expression in insulin-sensitive tissues may be a new strategy to increase insulin sensitivity and may also become a new target for the treatment of T2DM.

CDC42 and RAC1 are members of the Rho GTPase family, which regulate signaling pathways that control a variety of cellular functions, including cell morphology, migration, endocytosis, and cell cycle progression. Both CDC42 and RAC1 regulate the second phase of glucose-stimulated insulin secretion (GSIS), and the circulation of these proteins between the activated state (GTP-bound) and the inactive state (GDP-bound) is important for insulin secretion [13, 14].

CDC42 plays critical roles in the process of insulin synthesis by regulating granule fusion and cytoskeletal rearrangement [15, 16] and also regulates mobilization and cell membrane exocytosis and endocytosis of insulin granules via activating a series of downstream factors [17–20]. One study showed that upregulation of miR-330-3p reduces the expression of CDC42 and E2F1 in patients with gestational diabetes (GDM), resulting in impaired *β*-cell proliferation [21]. P21-activated kinase 1 (PAK1) is a downstream factor of CDC42 and an important promoter of cell proliferation. Another study showed an 80% reduction in PAK1 in patients with T2DM [2]. Thus, CDC42 is an important member in the progress of T2DM, and targeted therapy for CDC42 may be one of the effective methods for treating T2DM and related diseases.

RAC1, which can stimulate actin cytoskeleton reorganization [22], is required for insulin-stimulated translocation of glucose transporter 4 (GLUT-4) in muscle cells [23]. RAC1 also can activate PAK [24]. The study indicated that RAC1 and its downstream target protein PAK were reduced in insulin-resistant mice and human skeletal muscle [25]. In addition, RAC1 can activate NADPH oxygenase (NOX), which produces reactive oxygen species (ROS) and activates p38MAPK under high glucose conditions, leading to mitochondrial disorders and islet *β*-cell apoptosis [26, 27]. This mechanism also plays a crucial role in diabetes-induced vascular injuries, such as diabetic retinopathy [28] and diabetic cardiomyopathy [29]. Thus, RAC1 can be a novel molecular candidate of T2DM and provide new insight to improve therapeutic strategies for T2DM and diabetic complications.

GNG3, a member of signal-transducing molecules, a signal transduction molecule encoding the G protein gamma 3 subunit, plays a variety of roles during signal transduction, from membrane targeting of the *α* subunit [30] to receptor recognition [31], to activation of effectors [32], and then to effect signaling regulation of various proteins of intensity or duration [33]. The research found that inhibition of G-protein *βγ* signaling produces the changes in the cytokine mRNA levels, which can benefit the autoimmune diseases [34]. In addition, the mice lacking the G protein *γ*3 subtype show decreased weight gain, reduced fat intake, and defective Oprm1 signaling [35], when maintained on a high-fat diet. These results suggest that GNG3 may be involved in the pathogenesis of T2DM, and further research on GNG3 may provide new targets for the development of drugs to treat obesity and relevant diseases.

GNAI1, also known as Gi, an adenylate cyclase inhibitor that inhibits the conversion of ATP to cAMP [36], can interact with other proteins. T cell differentiation may change its structure [37]. Studies showed that altered expression of GNAI1 was associated with the progression of inflammation and immune disease [38, 39]. Thus, GNAII may be considered to be a novel biomarker for T2DM.

ITGB1, a member of the integrin family, consists of 18 *α* and 8 *β* transmembrane subunits that form at least 24 different heterodimeric receptors allowing cells to adhere to extracellular matrix (ECM) proteins [40]. Integrins play an important role in mediating cell-to-cell and cell-to-ECM adhesion [41], especially between the extracellular environment and platelets, inflammatory cells, and the vasculature [42]. The previous study has confirmed that integrin-mediated adhesion was preferentially mediated by ITGB1. Integrins have been shown to be involved in angiogenesis [43], which is a key pathological characteristic of diabetic microvascular complications and also is essential for homeostasis of adipose tissues. ITGB1 may be a therapeutic target for obesity [44]. Consistently, as a significant membrane gene identified in our study, ITGB1 was expressed differentially between T2DM and normal groups. ITGB1 may play central roles in all DEGs and have a close relationship with the development of obesity, T2DM, and its complications.

## 5. Conclusion

Our study tried to identify some candidate genes and pathway regulatory network closely related to T2DM by a series of bioinformatics analysis on DEGs between T2DM samples and normal samples. The findings in the current work may help us understand the underlying molecular mechanisms of T2DM. DEGs such as PIK3R1, RAC1, GNG3, GNAI1, CDC42, and ITGB1 have the potential to be used as targets for T2DM diagnosis and treatments. However, the lack of experimental validation is a limitation of this study. In the future, these prediction results obtained through bioinformatics analysis can be verified by further experimental studies such as qRT-PCR and Western blot.

## Figures and Tables

**Figure 1:** Cluster analysis of DEGs. The abscissa represents different samples; the vertical axis represents clusters of DEGs. Red indicates that expression of the gene is relatively upregulated while green indicates that expression of the gene is relatively downregulated; black indicates no significant changes in gene expression.

**Figure 2:** Enriched GO functions of DEGs. DEGs: differentially expressed genes; GO: Gene Ontology; BP: biological process; CC: cellular component; MF: molecular function.

**Figure 3:** KEGG pathway analysis of differentially expressed genes. KEGG: Kyoto Encyclopedia of Genes and Genomes.

**Figure 4:** Protein-protein interaction (PPI) networks constructed by STRING and modular analysis.

**Figure 5:** Venn diagram analysis of candidate genes. The blue circle represents core genes, the red circle represents hub genes, and the green circle represents bottleneck genes.

**Table 1:** The candidate genes selected from the protein-protein interaction network.

Core genes			Gene IDs
Cluster	Nodes	Edges	
1	15	104	AVPR1B CYSLTR2 EDN3 GHSR **GNG3** GRM5 KALRN LTB4R2 MLN NMBR NPFFR2 **PIK3R1** PTGFR SAA1 TBXA2R
2	13	78	ASB11 FBXL18 FBXL7 FBXO17 FBXO7 GLMN KLHL41 RNF7 UBE2H UBE2L6 UBE2V1 ZNF645 ZNRF1
3	8	28	CCL20 CXCL3 DRD2 **GNAI1** HRH4 NPY2R PTGER3 TAS2R46
4	8	28	ARMC8 CYFIP1 DEFA4 DNASE1L1 HP LTF OLFM4 VCL
5	8	28	CEACAM5 GP2 LY6G6C LY6H LY6K LYPD4 LYPD5 PRSS21
6	6	14	COL19A1 COL25A1 COL4A6 COL9A1 PLOD2 PPIB
7	5	10	CGA FSHB GLP2R GPR45 HTR4
8	10	22	APOA2 BCAR1 BMP4 EVA1A ITGB1 **ITGB3** MEN1 MET TMEM132A TNC
9	17	35	ARF6 BDNF **CDC42** CFTR FZD4 GBP6 GNAZ HLA-C HLA-DRB1 HLA-DRB5 ITSN2 NGFR NTRK2 **RAC1** SNX9 SYT9 TRIM62
Hub genes			AKT1 **CDC42** CREBBP **GNAI1 GNG3** GRM5 **ITGB1** KALRN **PIK3R1 RAC1** SAA1 TBXA2R
Bottleneck genes			AKT1 **CDC42** CEACAM8 CREBBP **GNAI1 GNG3 ITGB1** MAP2K3 **PIK3R1** PSMB8 **RAC1** RFC2 UBE2L6 UBE2V1

Candidate genes are shown in bold.

## Data Availability

The data used to support the findings of this study are available from the corresponding author upon request.
